This article has been retracted.

# Controlled Release of Curcumin from HPMC (Hydroxypropyl Methyl Cellulose) Co-Spray-Dried Materials

**DOI:** 10.1155/2021/7625585

**Published:** 2021-06-15

**Authors:** Jiao Zheng, Bo Wang, Jia Xiang, Zhengyu Yu

**Affiliations:** ^1^Drug Clinical Trial Institution Department, Hunan Provincial People's Hospital (The First Affiliated Hospital of Hunan Normal University), Changsha, Hunan 410000, China; ^2^Xiangya School of Pharmaceutical Sciences, Central South University, Changsha, Hunan 410000, China; ^3^Faculty of Engneering and IT, University of Technology, Sydney, NSW 2007, Australia

## Abstract

In order to achieve the controlled release of curcumin, HPMC (hydroxypropyl methyl cellulose) was spray dried with curcumin and lactose. The spray-dried materials were pressed into tablets with a diameter of 8 mm, and their release characteristics *in vitro* were measured. *In vitro* experiments showed that the release of curcumin from the HPMC mixture was significantly slower due to the sustained-release property of HPMC as a typical excipient. The release profile of curcumin from the HPMC mixture was relatively stable for a controlled release. SEM images show that the HPMC co-spray-dried powders have crumpled surfaces due to the large molecular weight of HPMC. DSC, XRD, FTIR, N_2_ adsorption, and TGA have been measured for the spray-dried curcumin materials. This work indicates that HPMC can be used as a controlled-release excipient for curcumin preparations.

## 1. Introduction

Curcumin is a hydrophobic polyphenol extracted from the root and stem of turmeric. It has a variety of pharmacological properties, including antioxidant, anti-inflammatory, anticancer, and treatment of nerve diseases [1]. However, curcumin is easily degraded by light induction and unstable under physiological pH of human body. In addition, its poor solubility in water leads to its low oral absorption efficiency and many challenges in clinical application [2]. Therefore, it is important to improve the chemical stability, solubility, and bioavailability of curcumin.

Hydroxypropyl methylcellulose (HPMC) is a semisynthetic dietary polymer based on cellulose. HPMC is used as a food ingredient and in the food industry as an emulsifier, suspension agent, film-forming agent, stabilizer, or thickener. In addition, HPMC is used as an excipient in pharmaceutical preparations to improve the solubility of active pharmaceutical ingredients and to control drug delivery [3–5].

Many methods have been reported to increase the solubility of curcumin and promote its bioavailability. Relative techniques include the preparation of colloids, protein-based complexes, solid dispersions, nanoemulsions [6–8], and so forth. However, most of these methods have complex processes and poor physical stability and many risks such as drug leakage and potential toxicity of excipients and reagents [6], which limits the clinical application.

Considering the physical product stability and security problems, the experimental design used water as a dispersion medium and selected lactose, a commonly used drug-excipient, as the water-soluble carrier. HPMC was used as the studying excipient for the control the curcumin dissolution rate. After high-speed stirring of mixed suspension, the spray drying technique was used to dry the mixture.

## 2. Materials and Methods

### 2.1. Chemicals

HPMC (SE-E5) was purchased from Anhui Sunhere Pharmaceutical Excipients Co., Ltd.; the pharmaceutical-grade *α*-lactose monohydrate (purity > 99.9%) was purchased from Jiangsu Dawning Pharmaceutical Co., Ltd.; and curcumin (purity > 98.0%) was purchased from Tonghua Food & Chemical Co., Ltd.

### 2.2. Design of the Experiment

In order to study the sustained-release effects of HPMC for curcumin, the experiment was carried out with spray drying of suspension A containing curcumin and lactose and suspension B containing curcumin, lactose, and HPMC, respectively. Suspension A contains 10% curcumin and 20% lactose in water, which were mixed at high stirring speed for 1 min. Suspension B contains 10% curcumin, 15% lactose, and 10% HPMC in water, after mixing by high-speed stirring, forming a foam-like mixture for spray drying. In the experiment, the same spray-drying parameters were used for the two suspensions. The spray dryer (YC-015A, Shanghai Pilotech Instrument & Equipment Co., Ltd.) was adjusted to the optimal parameters: an inlet air temperature of 140°C, outlet air temperature of 125°C, fan frequency of 50 Hz, peristaltic pump speed of 15 rpm/min, spray pressure of 0.65 MPa, and nozzle diameter of 1.0 mm. Suspensions A and B were spray dried, respectively, and the powders were collected in the collection vessel [9].

### 2.3. Characterization of the Spray-Dried Materials

The UV-vis absorption spectra were recorded in the range 350–450 nm [10] with a UV-2401PC spectrophotometer (Shimadzu, Kyoto, Japan). The powder was pressed into tablets with a diameter of 8 mm and then dissolved in pure water; both samples were prepared in triplicate at room temperature. DSC analysis was performed using a differential scanning calorimeter (HSC-4 DSC, Henven, China) for the solid powder. The sample for DSC measurement was prepared following standard procedures using a sealed aluminum pan. About 10 mg of sample was used in the analysis. The analyses were performed by heating the samples from 25°C to 300°C at a heating rate of 5°C/min with N_2_ as the purge gas. Heat flow as a function of increasing temperature was recorded for the analysis of each sample. Fourier transform infrared (FTIR) spectroscopy was used to investigate the production and the raw material (HPMC, lactose, and curcumin crystle). The specimen was mixed with KBr powder, tableted, and scanned for transmission sensitivity in a Nicolet 6700 FTIR spectrometer (Thermo Fisher Scientific). The FTIR spectra used a resolution of 1 cm^−1^ with 64 scans. The solid powder sample was placed on a carbon tape on an aluminum sample spike. The gold-plated particles were observed by using a JSM-7200F scanning electron microscope (SEM, JEOL Ltd.). Thermogravimetric analysis (TGA Q5000 V3.17 Build 265) was performed for the sample. Measurement was carried out on the sample loaded in small alumina pans with N_2_ as the balance gas. The temperature was set from 20°C to 350°C, with a constant heating rate of 5°C/min, under a flow of nitrogen gas in pyrolysis condition. XRD analysis was used to investigate the crystalline characteristics of the solid powder. Solid samples were loaded on powder holders and analyzed using a Siemens D5000 diffractometer. One gram of the sample was dispersed in the sample holder. The scanning region of diffraction angle (2*θ*) was set from 5 to 40° with a scanning rate of 1.2°/min, a scanning current of 30 mA, and a scanning voltage of 40 kV. The N_2_ adsorption was carried out for the powder sample to determine the porosity.

### 2.4. Results and Discussion

Figure 1 shows the release profiles of curcumin for the HMPC and non-HMPC tablets under the same conditions. The spray drying of curcumin with lactose has an obvious effect on promoting its dissolution, where 90% of curcumin was released in 10 min. When HPMC was added, the release of curcumin was gradually increased with 90% released in 40 min. The sustained-release property of HPMC can avoid a sudden release of API (active pharmaceutical ingredient) after the drug entering the human body, possibly benefiting the bioavailability.

In order to further study the HPMC effect in a microsense, scanning electron microscopy (SEM) was used. As shown in Figures 2(a) and 2(b), the spray-dried materials from suspension A (curcumin and lactose) are uniform spheres, where curcumin was microencapsulated in a lactose excipient. However, for the solid powder mixture obtained from suspension B (HMPC contained), the surface of the spray-dried powder is crumpled as shown in Figures 2(c) and 2(d). The crumpled surfaces were possibly caused by the coating of HPMC which had a high molecular weight. The large molecules have low diffusion coefficient in water during spray drying and remained on the surfaces after drying. In addition, HPMC can form hydrogen bonds with curcumin befitting the release and permeability [11].

The DSC curves (Figure 3) show that the HPMC-contained sample has an upward exothermic peak at 210–220°C, indicating the mixing of these materials. Besides, the HPMC-contained sample has a large endothermic peak of free water at 50–100°C, suggesting that the HPMC bonded some water molecules. Some small peaks are observed, which may indicate the formation of a relatively more disordered crystalline state [11]. According to the XRD spectrum of the HPMC-contained sample (Figure 4), *α*-lactose peaks are observed at 2*θ* of 12.5°, 19.1°, 19.6°, and 19.9°. The spectra showed that the HPMC-contained sample was crystalline with sharp peaks observed. The changes in peak intensity and wavenumber shift were studied by FTIR (Figure 5). The peak of 3400 cm^−1^ indicates the presence of hydroxide, indicating the presence of water which agreed with the DSC result [12, 13].

BET (Figure 6) spectra show the N_2_ adsorption-desorption isotherms for the HPMC-contained sample. The isotherms display class II behavior. In the process of increasing gas pressure, countermolecular layer adsorption and multimolecular layer adsorption are carried out simultaneously in which the “knee” point is not sharp. According to the BET result, the sample has a nonporous or macroporous structure. According to TGA analysis (Figure 7), HPMC did not affect much on the result since the polymer has a large molecular weight.

## 3. Results

In this work, HPMC was spray dried with curcumin and lactose. The spray-dried materials were pressed into tablets, and its release characteristics *in vitro* were measured. *In vitro* experiments showed that the release of curcumin from the HPMC mixture was significantly slower due to the sustained-release property of HPMC as a typical excipient. The release profile of curcumin from the HPMC mixture was relatively stable for a controlled release. SEM images show that the HPMC co-spray-dried powders have crumpled surfaces due to the large molecular weight of HPMC. DSC, XRD, FTIR, N_2_ adsorption, and TGA have been measured for the spray-dried curcumin materials. The work indicates that HPMC can be used as a controlled-release excipient for curcumin preparations.

## Figures and Tables

**Figure 1:** Release profiles of curcumin from the HMPC and non-HMPC tablets.

**Figure 2:** SEM images of the spray-dried non-HPMC (a and b) and HPMC materials (c and d), obtained from suspension A and B, respectively.

**Figure 3:** DSC spectrum of the raw materials and productions.

**Figure 4:** XRD spectrum of the HPMC-contained sample.

**Figure 5:** FTIR spectra of the products and the raw materials.

**Figure 6:** The N_2_ adsorption and desorption curves of the HPMC-contained sample.

**Figure 7:** The TGA curve of the spray-dried non-HMPC and HPMC-contained materials.

## Data Availability

All data used to support the findings of this study are included within the article.
